# Applying the Fuzzy Analytic Hierarchy Process Method to Evaluate Key Indicators of Health Promotion Policies for the Elderly in Taiwan

**DOI:** 10.1155/2021/4832877

**Published:** 2021-11-18

**Authors:** Ling-Mei Hsu, Ji-Feng Ding

**Affiliations:** ^1^Program in Business and Operations Management, Chang Jung Christian University, Tainan City 71101, Taiwan; ^2^Department of Aviation and Maritime Transportation Management, Chang Jung Christian University, Tainan City 71101, Taiwan

## Abstract

Investigation of the key indicators of health promotion policies for an aging society can shed light on the priority of the government's health promotion efforts. This study applied the fuzzy analytic hierarchy process (AHP) method in an empirical analysis of the key indicators of the health promotion policies for Taiwan's aging society. Based on a review of the literature and expert interviews, this paper first conducted a preliminary study and evaluation of major factors affecting health promotion policies and found 4 major evaluation aspects and 16 evaluation indicators. After employing an AHP expert questionnaire in an empirical investigation, the following findings were made: (1) “healthy living” was the most important evaluation aspect for Taiwan's health promotion policies for its aging society. (2) The six leading key indicators of health promotion policies were “promotion of personal health awareness and behavior,” “promotion of home medical services,” “guaranteeing the economic security of the elderly,” “planning a family caregiver support service system,” “well-planned health promotion plans for the elderly,” and “training long-term care service personnel and providing professional medical care.” Following discussion, recommendations concerning these six key indicators are made as a reference for future evaluation of health promotion policies for an aging society.

## 1. Introduction

Taiwan's population over the age of 65 has accounted for more than 14% of the total population since 2018, which indicates that Taiwan has become an aging society [1]. According to the estimates of Taiwan's National Development Council, the proportion of people over 65 years old will exceed 20% by 2025, implying that 1 out of every 5 people will be an older person and making Taiwan a superaged society [2]. Taiwan is already one of the countries with the fastest rate of aging in the world [3]. This trend shows that Taiwan must face the challenge of demographic aging. With the approach of a superaged society, various government ministries have been reviewing and cooperating on issues concerning policies for the elderly. The development of effective health promotion for an aging society is one of the government's core policies, and it is believed that sound health promotion policies can effectively reduce the health risks and medical costs of the elderly and improve their quality of life.

At present, the leading countries of Europe, America, and Japan are facing the problem of a declining birthrate and aging population, and progress in medicine and public health has increased average life expectancy. As a consequence, issues connected with an aging society (such as health and well-being issues) are attracting growing attention from these countries' governments [4, 5]. According to the estimates of the World Health Organization (WHO), the growth rate of the world's elderly population will be as high as 223% in 2025. By 2025, 80% of the elderly are expected to suffer from at least one chronic disease, and 50% of the elderly will suffer from two or more chronic diseases [6]. The treatment of chronic diseases of the elderly will account for 66% of the medical budget [7, 8]. These projections indicate that the medical costs of an aging society will be high. However, research has also shown that the implementation of health promotion plans can effectively reduce health risks and healthcare costs for the elderly [9]. The governments of various countries are therefore paying increasing attention to health promotion and care for the elderly.

The 1st International Conference on Health Promotion was held by the WHO in Ottawa, Canada, in 1986 and formulated the “Ottawa Charter for Health Promotion 1986.” This event achieved a consensus that health promotion should be a process of empowering people and enabling them to improve their health [10]. Green and Kreuter [11] proposed that health promotion is the systematic combination of educational, political, legal, and organizational support in strategies for strengthening individuals' health. The WHO defines health promotion as a process of enabling people to strengthen and improve control of their health [12]. The WHO also advocates the concept of “active aging,” which seeks that life can be prolonged with a healthy lifestyle into a dignified old age [13]. In an aging society, the concept of “active aging” that can enable the elderly to autonomously control health-related activities has become a central focus of policy development.

The government of Taiwan will face severe challenges from an aging and superaged society in the near future. As a consequence, the government is actively pursuing the development of health promotion policies for the elderly. However, whether the content of the government's health promotion policies meets elderly citizens' health promotion needs remains an important policy evaluation issue. Investigating the development factors of health promotion in an aging society will help shed light on what the elderly need from health promotion policies. In addition, the findings of this investigation will also suggest how the government should prioritize measures related to health promotion in light of its limited resources. As a result, the evaluation of whether the developmental elements of Taiwan's health promotion policies meet the needs of the elderly and assessment of the government's policy performance in instituting health promotion policies are consequently research topics deserving of exploration in depth.

The development of health promotion policies for an aging society involves numerous factors, and criteria and indicators constitute important standards to guide decision-making in this type of situation [14]. How a decision-maker should decide which indicators should be assigned the weights when promoting health policies is thus an important matter. In the multiple criteria decision-making (MCDM) assessment process, the construction of an objective hierarchical structure through hierarchy analysis is a key step [15]. When a hierarchical framework of relationships has been established, it will make the decision-making assessment questions clearer and more concrete, making the decision-makers' task much easier. Accordingly, this study employed this method to preliminarily draft indicators for the assessment of the development of health promotion policies for Taiwan's aging society. These preliminary indicators are based on the policies and experience of advanced countries [16] and the health promotion model (HPM) [17] and refer to the policy blueprint for aging society by the Ministry of Health and Welfare (MOHW) of Taiwan [18]. Because the research scope and levels involved in the evaluation of health promotion for an aging society are wide and complex, this process can be effectively tackled employing MCDM [14, 19]. The analytic hierarchy process (AHP) [15] is a set of decision-making methods for systematically solving complex problems and is chiefly used in uncertain situations and decision-making problems with multiple attributes. This study therefore used the AHP method to assess the relative importance of health promotion development indicators. However, the various health promotion development indicators have qualitative characteristics, and the weights expressing the importance of these indicators may be ambiguous in different situations [20–22]. Because an evaluator's subjective assessment of an indicator will therefore have fuzzy characteristics [22], it will be difficult to express the importance of key health promotion policies indicators with precise numerical values. In light of these circumstances, this study consequently applied fuzzy set theory [22] in conjunction with the AHP method to construct a fuzzy AHP evaluation model. This model was then used to evaluate the key indicators of health promotion policies for an aging society.

In summary, to address the needs of Taiwan's aging society, the MOHW must propose a comprehensive and effective health promotion policy blueprint. To ensure that policy assessment reflects the health promotion development needs of older adults, this paper employed a systematic, scientific empirical assessment to gain a better understanding of the key performance indicators of the government's health promotion policies. This assessment involved the application of the fuzzy AHP method to empirically analyze the key indicators of the development of health promotion policies for an aging society in Taiwan. It is hoped that the results of this paper can provide a reference for future evaluation of health promotion policies for an aged society. This study's contribution was therefore the use of the AHP method and an expert questionnaire to perform the empirical assessment of key indicators of Taiwan's health promotion policies. The findings obtained from this process can guide the government's use of policy indicators and strategies and can enable a better response to the health promotion needs of the coming superaged society. It is also worth noting that the fuzzy AHP assessment model developed in this paper can be employed as a practical tool for business applications. Particularly in ambiguous situations, this model can be developed as a decision-making support system helping users to assess decision-making questions. Apart from this section, Section 2 of this paper reviews relevant literature, Section 3 introduces research methods, Section 4 conducts empirical analysis and discussion, and Section 5 puts forth conclusions.

## 2. Literature Review

Demographic aging has now become a global phenomenon. Because human physical functions gradually deteriorate with age [4, 5], the health and long-term care of the elderly have become focal points for the governments of many countries [3]. Since Taiwan became an aging society, the government has been paying increasing attention to the health problems of older adults [2, 3] and seeks to help the elderly live healthier and have a better quality of life. As a result, the development of health promotion policies for the elderly has become one of the government's governance priorities [10, 12].

Although medical advances have prolonged the human lifespan, they have neither solved many of the health problems faced by older adults nor necessarily improved their quality of life [23, 24]. Healthcare, health promotion, and preventive healthcare are therefore all key issues [5]. The health promotion model proposed by Pender et al. [17] is currently the most common model used to guide health promotion for the elderly. This model chiefly explores which factors will induce older individuals to engage in health-promoting physical, psychological, and social behaviors. The model also takes into consideration that individuals' awareness of expected behavioral benefits and obstacles will directly affect their health-promoting behaviors. The “Ottawa Charter for Health Promotion” proposed by WHO defines health promotion as a process enabling people to control the determining factors of their health and thereby improve their health [10, 25–28]. The scope of health promotion for older adults encompasses proper nutrition, sports and leisure, stress management, health responsibility, self-realization, and the development of social support systems [25]. This implies that health promotion for the elderly is not limited to the treatment and alleviation of diseases and disabilities. Instead, it should seek to promote the overall health of the body, mind, and spirit while extending the lifespan and reducing deaths among older adults. Older adults should have a sense of well-being, a comfortable life, and the ability to actively enjoy a “happy and joyful” life in old age [29]. Health promotion should therefore stimulate the full potential of older adults, reduce the impacts of aging, and improve the quality and value of their life [24, 29].

The European Union (EU) has proposed the concept of active aging, which refers to various strategies that can be used to extend life, improve health, and strengthen personal and social resources. In practice, active aging chiefly includes helping the elderly attain a healthier lifestyle, extend their working life, delay their retirement, and maintain an active life after retirement [30]. The EU has also proposed a health promotion plan containing recommendations concerning the drafting of national health aging policies. These policies should be in accord with the social values of older adults and comply with the health promotion principle of necessity, equality, autonomy, and specificity [16, 24, 30].

The main purpose of the health promotion policies issued by the US government is to extend people's lives and improve their quality of life, thereby making the American people healthier [31]. The purpose of the Older Americans Act [32–37] is to assist the independent living of the elderly at home and provide transportation assistance and home safety care. Community-based services include daytime care for the elderly, assistance through referral services, and community activity centers. Food and nutrition services chiefly consisting of meal delivery allow the elderly to enjoy food and avoid hunger. The emphasis on health prevention services mainly attempts to promote a healthy lifestyle for the elderly through physical exercise, a balanced diet, regular health checks, and the provision of various health education activities in their daily lives.

The United Kingdom proposed a ten-year plan for the integration of national services for older adults [38]. The goal of this plan is to eliminate discrimination against the elderly, promote the health and independence of the elderly, and meet the health needs of the elderly. British health promotion strategies for older adults include individual-centered care services, intermediate care medical care, prevention of stroke and falls, mental health consultation for the elderly, and active aging life.

Japan has proposed the “Healthy Japan 21” health program [39], which calls for the establishment of a healthy environment in the initial prevention stage, setting of goals and evaluation of results, and cooperation among relevant agencies in the formulation and implementation of effective health promotion activities. With a focus on living habits and diseases, the program emphasizes the development of health promotion strategies for older adults by the country as a whole, with the joint participation of industry, government, and academia.

Taiwan has issued the “White Paper on Aging Society” [18, 40], which takes health promotion as its core spirit. The White Paper's goal is to build a healthy aging society, happy families, a vibrant society, and a friendly environment, and it seeks to establish a new blueprint for health promotion in Taiwan's aging society.

In order to obtain performance indicators for health promotion policies, this study first summarized health promotion content proposed by governments and scholars and assembled the preliminary health promotion policy development indicators shown in Table 1.

In AHP, the first task is to determine the hierarchical structure of the system in question [15], and this structure is then used to study the interactions of various elements and their impact on the system as a whole. The number of elements in the hierarchy depends on the complexity of the system and analytical needs. Too many evaluation indicators or criteria will increase the evaluation time and cost. On the other hand, if there are too few indicators or criteria, the quality of content and applicability of the evaluation criteria cannot be clearly determined. Hence, the establishment of a set of evaluation indicators or criteria with a clearly defined hierarchical structure is an important task when using the AHP approach.

In general, the drafting of criteria must comply with five principles, namely, completeness, operational, decomposable, nonredundancy, and minimum size [15]. Indicators should typically be specific, observable, and measurable accomplishments and should constitute standards for assessment of whether the specific desired outcome can be achieved. The indicators chosen by researchers must be able to answer the assessment questions being asked and must help the researchers determine whether the goal of their questions has been achieved [14, 15, 19]. In order to establish an objective hierarchical structure, this study first conducted a review of the literature concerning factors influencing health promotion policies. The next step was to involve relevant stakeholders in the process of brainstorming in order to develop a set of assessment indicators. To obtain preliminary indicators of Taiwan's health promotion policies, the indicators in Table 1 were reviewed and discussed by five scholars and experts with over 20 years of experience. As a result, the four chief assessment aspects of health promotion policies for Taiwan's aging society of healthy living, family well-being, a vibrant society, and a friendly environment were obtained; the 16 major indicators under these aspects and a description of their features can be seen in Table 2.

## 3. Research Methods

This section is a brief description of the triangular fuzzy number and its arithmetic operations, ranking of the triangular fuzzy number, and the fuzzy AHP method.

### 3.1. Triangular Fuzzy Number and Its Arithmetic Operations

Let *X* be a set of things, which is called a universal set (or universe of discourse). For a universal set *X* and the functions $\mu_{\tilde{A}}:X⟶\left[0,1\right]$ defined on it, the set $\tilde{A}=\left\{\left(x,\mu_{\tilde{A}}\left(x\right)\right)|x\in X\right\}$ is called a fuzzy subset on *X*, $\mu_{\tilde{A}}\left(x\right)$ is called the grade of membership of *x* in $\tilde{A}$ , and $\mu_{\tilde{A}}$ is called the membership function of $\tilde{A}$ . The closer the value of $\mu_{\tilde{A}}\left(x\right)$ is to 1, the higher the degree of membership of *x* in $\tilde{A}$.

If there is a fuzzy number $\tilde{A}$ [41], suppose its membership function $\mu_{\tilde{A}}:ℜ⟶\left[0,1\right]$, as shown in equation (1):

(1) $$\begin{array}{c} \mu_{\tilde{A}}\left(x\right)=\left\{\begin{array}{cc} \frac{\left(x-a\right)}{\left(b-a\right)}, & a\leq x\leq b\\ \frac{\left(x-c\right)}{\left(b-c\right)}, & b\leq x\leq c\\ 0, & \text{otherwise} \end{array},\right. \end{array}$$

where −*∞* < *a* ≤ *b* ≤ *c* < *∞*; the fuzzy number is called the triangular fuzzy number. The triangular fuzzy number $\tilde{A}$ is expressed with (*a*, *b*, *c*) as $\tilde{A}=\left(a,b,c\right)$.

According to Zadeh's extension principle [22], assuming ${\tilde{A}}_{1}=\left(a_{1},b_{1},c_{1}\right)$ and ${\tilde{A}}_{2}=\left(a_{2},b_{2},c_{2}\right)$, the following fuzzy expressions are always true:

(1) Fuzzy addition:
  (2) $$\begin{array}{c} {\tilde{A}}_{1}⊕{\tilde{A}}_{2}=\left(a_{1}+a_{2},b_{1}+b_{2},c_{1}+c_{2}\right). \end{array}$$
(2) Fuzzy subtraction:
  (3) $$\begin{array}{c} {\tilde{A}}_{1}\Theta {\tilde{A}}_{2}=\left(a_{1}-c_{2},b_{1}-b_{2},c_{1}-a_{2}\right). \end{array}$$
(3) Fuzzy multiplication:
  (4) $$\begin{array}{c} k⊗\tilde{A}=\left(\mathrm{ka,}\;\mathrm{kb,}\;\mathrm{kc}\right),\;k\geq 0,\;k\in R;\\ {\tilde{A}}_{1}⊗{\tilde{A}}_{2}≅\left(a_{1}a_{2},b_{1}b_{2},c_{1}c_{2}\right)\;\mathrm{If}\;a_{1}\geq 0\;a_{2}\geq 0. \end{array}$$
(4) Fuzzy division:
  (5) $$\begin{array}{c} {\left({\tilde{A}}_{1}\right)}^{-1}≅\left(\frac{1}{c_{1}},\frac{1}{b_{1}},\frac{1}{a_{1}}\right),a_{1}>0,\\ {\tilde{A}}_{1}\;\emptyset \;{\tilde{A}}_{2}≅\left(\frac{a_{1}}{c_{2}},\frac{b_{1}}{b_{2}},\frac{c_{1}}{a_{2}}\right)\;\text{if }a_{1}\geq 0,a_{2}>0. \end{array}$$
(5) Fuzzy *k*^th^ root:
  (6) $$\begin{array}{c} {\left({\tilde{A}}_{1}\right)}^{1/k}≅\left(a_{1}^{1/k},b_{1}^{1/k},c_{1}^{1/k}\right),a_{1}\geq 0,k\geq 2. \end{array}$$

### 3.2. Ranking of Triangular Fuzzy Numbers

Scholars have done researches on the methods of ranking fuzzy numbers. Chen and Hsieh [42] put forward a graded mean integration representation (GMIR) after comparing various methods. This paper has adopted the GMIR method to solve the problem of defuzziness calculation of ranking fuzzy numbers.

According to the GMIR method proposed by Chen and Hsieh, let ${\tilde{A}}_{i}=\left(a_{i},b_{i},c_{i}\right)$, *i*=1,2,…, *n*, be *n* triangular fuzzy numbers. The GMIR value of the triangular fuzzy number ${\tilde{A}}_{i}$ can be expressed as $G\left({\tilde{A}}_{i}\right)$

(7) $$\begin{array}{c} G\left({\tilde{A}}_{i}\right)=\frac{a_{i}+4b_{i}+c_{i}}{6}. \end{array}$$

This paper defined the ranking rules of two fuzzy numbers ${\tilde{A}}_{i}$ and ${\tilde{A}}_{j}$ as follows:

1. ${\tilde{A}}_{i}>{\tilde{A}}_{j}\Leftrightarrow G\left({\tilde{A}}_{i}\right)>G\left({\tilde{A}}_{j}\right)$.
2. ${\tilde{A}}_{i}<{\tilde{A}}_{j}\Leftrightarrow G\left({\tilde{A}}_{i}\right)<G\left({\tilde{A}}_{j}\right)$.
3. ${\tilde{A}}_{i}<{\tilde{A}}_{j}\Leftrightarrow G\left({\tilde{A}}_{i}\right)<G\left({\tilde{A}}_{j}\right)$.

### 3.3. Fuzzy AHP Method

AHP [15] is an MCDM method proposed during the 1970s by Professor Thomas Saaty at the University of Pennsylvania and subsequently developed at the University of Pittsburgh. Buckley [43] extended hierarchical analysis using a consistency test method for fuzzy positive reciprocal matrices in which all elements are trapezoidal fuzzy numbers. Buckley et al. [44] later revisited fuzzy hierarchical analysis and proposed a new method of finding fuzzy weights. Since that time, research involving the use of the fuzzy AHP method has appeared in countless academic journals, and the method has been applied to a vast number of MCDM problems [45–53]. This paper chiefly referred to the methods of Hsu [54] and Ding et al. [55] regarding the fuzzy AHP method. A brief description of the steps used in the fuzzy AHP method in this paper is as follows.

Step 1: Establishing a hierarchical structure.
This paper used Figure 1 as the hierarchical structure diagram. In this structure, the *L* layer is the problem, that is, to obtain the key indicators of the health promotion policies in Taiwan for an aging society. At the L + 1 layer, *k* is an evaluation aspect. The L + 2 layer is the evaluation indicator *p*+⋯+*q*+⋯+*r* under each evaluation aspect.
Step 2: Establishing crisp values for pairwise comparison.
The pairwise comparison questionnaires are used to obtain experts' opinions on the relative importance of the two evaluation indicators (as shown in Table 3).
  (1) Set *x*_*ij*_^*E*^ as the view of an expert *E*, *E*=1,2,…, *h*, of the relative importance of any two evaluation aspects *i* and *j* in the *L* + 1 layer. Then a pairwise comparison matrix in the *L* + 1 layer is [*x*_*ij*_^*E*^]_*k*×*k*_.
  (2) Set *x*_*fg*_^*E*^ as the view of an expert *E*, *E*=1,2,…, *h*, of the relative importance of any two evaluation indicators *f* and *g* in the corresponding *L* + 2 layer under a certain evaluation aspect of *C*_1_^*L*+1^, *C*_*t*_^*L*+1^, and *C*_*k*_^*L*+1^ of the *L* + 1 layer. Then the pairwise comparison matrices of the evaluation indicators in the *L* + 2 layer are [*x*_*fg*_^*E*^]_*p*×*p*_, [*x*_*fg*_^*E*^]_*q*×*q*_, and [*x*_*fg*_^*E*^]_*r*×*r*_, respectively.
Step 3: Establishing triangular fuzzy numbers.
To integrate the consensus of experts [15, 54, 56], this paper takes the minimum evaluation value of a certain criterion by the decision-making members as the lower bound of the triangular fuzzy number. The maximum evaluation value is taken as the upper bound of the triangular fuzzy number. The geometric mean of all evaluation values is regarded as 1 value for the grade of membership of the triangular fuzzy numbers.
Set *x*_*ij*_^*E*^ ∈ [1/9, 1/8,…, 1/2, 1] ∪ [1,2,…, 8,9], as the view of an expert *E*, *E*=1,2,…, *h*, of the relative importance of any two evaluation aspects *i* and *j*, ∀*i*, *j*=1,2,…, *k*, in the *L* + 1 layer, and then ${\tilde{A}}_{ij}^{L+1}=\left(a_{ij},b_{ij},c_{ij}\right)$ is the triangular fuzzy number after integration of all *h* experts in the *L* + 1 layer, where
  (8) $$\begin{array}{c} a_{ij}=\min\left\{x_{ij}^{1},x_{ij}^{2},\ldots ,x_{ij}^{h}\right\},\\ b_{ij}={\left(\prod_{E=1}^{h}x_{ij}^{E}\right)}^{1/h},\\ c_{ij}=\max\left\{x_{ij}^{1},x_{ij}^{2},\ldots ,x_{ij}^{h}\right\}. \end{array}$$
Similarly, for any two evaluation indicators in the *L*+2 layer, the triangle fuzzy number after integration is ${\tilde{A}}_{fg}^{L+2}=\left(a_{fg},b_{fg},c_{fg}\right),$∀*f*, *g*=1,…, *p*; ⋯; ∀*f*, *g*=1,…, *q*; ⋯; ∀*f*, *g*=1,…, *r*, where
  (9) $$\begin{array}{c} a_{fg}=\min\left\{x_{fg}^{1},x_{fg}^{2},\ldots ,x_{fg}^{h}\right\},\\ b_{fg}={\left(\prod_{E=1}^{h}x_{fg}^{E}\right)}^{1/h},\\ c_{fg}=\max\left\{x_{fg}^{1},x_{fg}^{2},\ldots ,x_{fg}^{h}\right\}. \end{array}$$
Step 4: Establishing the fuzzy positive reciprocal matrix of each layer.
For the integrated fuzzy number after the pairwise comparison of all experts at each layer, a fuzzy positive reciprocal matrix is established. For the *L* + 1 layer (the evaluation aspect layer), the fuzzy positive reciprocal matrix is
  (10) $$\begin{array}{c} A_{k}^{L+1}={\left[{\tilde{A}}_{ij}^{L+1}\right]}_{k\times k}=\left[\begin{array}{cccc} \tilde{1} & {\tilde{A}}_{12}^{L+1} & \cdots & {\tilde{A}}_{1k}^{L+1}\\ \frac{1}{{\tilde{A}}_{12}^{L+1}} & \tilde{1} & \cdots & {\tilde{A}}_{2k}^{L+1}\\ \vdots & \vdots & \ddots & \vdots \\ \frac{1}{{\tilde{A}}_{1k}^{L+1}} & \frac{1}{{\tilde{A}}_{2k}^{L+1}} & \cdots & \tilde{1} \end{array}\right],\text{where}\;{\tilde{A}}_{ij}^{L+1}⊗{\tilde{A}}_{ji}^{L+1}≅1,\;\forall i,\;j=1,2,\ldots ,k. \end{array}$$
In the same way, it can be analogized in the *L* + 2 layer. That is, as far as the *L* + 2 layer (evaluation indicator layer) is concerned, its fuzzy positive reciprocal matrix can be expressed as
  (11) $$\begin{array}{c} B_{p}^{L+2}={\left[{\tilde{B}}_{fg}^{L+2}\right]}_{p\times p}=\left[\begin{array}{cccc} \tilde{1} & {\tilde{B}}_{12}^{L+2} & \cdots & {\tilde{B}}_{1p}^{L+2}\\ \frac{1}{{\tilde{B}}_{12}^{L+2}} & \tilde{1} & \cdots & {\tilde{B}}_{2p}^{L+2}\\ \vdots & \vdots & \ddots & \vdots \\ \frac{1}{{\tilde{B}}_{1p}^{L+2}} & \frac{1}{{\tilde{B}}_{2p}^{L+2}} & \cdots & \tilde{1} \end{array}\right], \end{array}$$
where ${\tilde{B}}_{fg}^{L+2}⊗{\tilde{B}}_{gf}^{L+2}=1,\;\forall f,g=1,2,\ldots ,p$,……,
  (12) $$\begin{array}{c} B_{q}^{L+2}={\left[{\tilde{B}}_{fg}^{L+2}\right]}_{q\times q}=\left[\begin{array}{cccc} \tilde{1} & {\tilde{B}}_{12}^{L+2} & \cdots & {\tilde{B}}_{1q}^{L+2}\\ 1/{\tilde{B}}_{12}^{L+2} & \tilde{1} & \cdots & {\tilde{B}}_{2q}^{L+2}\\ \vdots & \vdots & \ddots & \vdots \\ 1/{\tilde{B}}_{1q}^{L+2} & 1/{\tilde{B}}_{2q}^{L+2} & \cdots & \tilde{1} \end{array}\right], \end{array}$$
where ${\tilde{B}}_{fg}^{L+2}⊗{\tilde{B}}_{gf}^{L+2}=1,\;\forall f,g=1,2,\ldots ,q$, and
  (13) $$\begin{array}{c} B_{r}^{L+2}={\left[{\tilde{B}}_{fg}^{L+2}\right]}_{r\times r}=\left[\begin{array}{cccc} \tilde{1} & {\tilde{B}}_{12}^{L+2} & \cdots & {\tilde{B}}_{1r}^{L+2}\\ 1/{\tilde{B}}_{12}^{L+2} & \tilde{1} & \cdots & {\tilde{B}}_{2r}^{L+2}\\ \vdots & \vdots & \ddots & \vdots \\ 1/{\tilde{B}}_{1r}^{L+2} & 1/{\tilde{B}}_{2r}^{L+2} & \cdots & \tilde{1} \end{array}\right], \end{array}$$
where ${\tilde{B}}_{fg}^{L+2}⊗{\tilde{B}}_{gf}^{L+2}=1,\;\forall f,g=1,2,\ldots ,r.$
Step 5: Calculating the fuzzy weight of fuzzy positive reciprocal matrix of each layer.
For the *L* + 1 layer, set ${\tilde{Z}}_{i}^{L+1}≅{\left({\tilde{A}}_{i1}^{L+1}⊗{\tilde{A}}_{i2}^{L+1}⊗\cdots ⊗{\tilde{A}}_{ik}^{L+1}\right)}^{1/k},\forall i=1,2,\ldots ,k,$ as the geometric mean of the triangular fuzzy numbers of the *i-*th evaluation aspect; then the fuzzy weight of the *i-*th evaluation aspect can be expressed as
  (14) $$\begin{array}{c} {\tilde{W}}_{i}^{L+1}≅{\tilde{Z}}_{i}^{L+1}⊗{\left({\tilde{Z}}_{1}^{L+1}⊕{\tilde{Z}}_{2}^{L+1}⊕\cdots ⊕{\tilde{Z}}_{k}^{L+1}\right)}^{-1}. \end{array}$$
For the convenience of symbol representation, the triangular fuzzy number is represented by ${\tilde{W}}_{i}^{L+1}=\left(w_{i}^{a},w_{i}^{b},w_{i}^{c}\right)$.
In the same way, any two evaluation indicators in the *L* + 2 layer can be deduced by analogy. That is, set ${\tilde{Z}}_{f}^{L+2}≅{\left({\tilde{B}}_{f1}^{L+2}⊗{\tilde{B}}_{f2}^{L+2}⊗\cdots ⊗{\tilde{B}}_{fp}^{L+2}\right)}^{1/p},\forall f=1,2,\ldots ,p,$ as the geometric mean of the triangular fuzzy numbers of the *f-th* evaluation indicator; then the fuzzy weight of the *f-*th evaluation indicator can be expressed as
  (15) $$\begin{array}{c} {\tilde{W}}_{f}^{L+2}≅{\tilde{Z}}_{f}^{L+2}⊗{\left({\tilde{Z}}_{1}^{L+2}⊕{\tilde{Z}}_{2}^{L+2}⊕\cdots ⊕{\tilde{Z}}_{p}^{L+2}\right)}^{-1}. \end{array}$$
For the convenience of symbol representation, the triangular fuzzy number is represented by ${\tilde{W}}_{f}^{L+2}=\left(w_{f}^{a},w_{f}^{b},w_{f}^{c}\right)$.
To save space, the fuzzy weights of other evaluation indicators [(*p*+⋯+*q*+⋯+*r*) − *p*] in the *L* + 2 layer can also be obtained by the above method.
Step 6: Defuzzifying the fuzzy weights.
This paper used the GMIR method proposed by Chen and Hsieh to defuzzify [42] the fuzzy numbers. The reason is that, in the process of defuzzification, Chen and Hsieh's method is more effective and easier to use.
Let ${\tilde{W}}_{i}^{L+1}=\left(w_{i}^{a},w_{i}^{b},w_{i}^{c}\right)$, ∀*i*=1,2,…, *k*, be a triangular fuzzy weight; then the *k-*th crisp weight after defuzzification is
  (16) $$\begin{array}{c} G\left({\tilde{W}}_{i}^{L+1}\right)=\frac{w_{i}^{a}+4w_{i}^{b}+w_{i}^{c}}{6},\forall i=1,2,\ldots ,k. \end{array}$$
The same is analogized for the *L* + 2 layer.
Step 7: Normalizing the crisp weights.
To facilitate the comparison of the relative importance of the evaluation aspects and the evaluation indicators at each layer, it is planned to normalize the *k-*th crisp weight after the abovementioned defuzzification as
  (17) $$\begin{array}{c} NW_{i}^{L+1}=\frac{G\left({\tilde{W}}_{i}^{L+1}\right)}{\sum_{i=1}^{k}G\left({\tilde{W}}_{i}^{L+1}\right)}. \end{array}$$
Step 8: Calculating the integrated weights of each evaluation criterion.
Suppose that the normalized crisp weights of the *L* + 1 layer and the *L* + 2 layer are represented by *NW*_*i*_^*L*+1^(∀*i*=1,2,…, *k*) and *NW*_*f*_^*L*+2^(∀*f*=1,…, *p*; ⋯; ∀*f*=1,…, *q*; ⋯; ∀*f*=1,…, *r*), respectively; then
  (1) The integrated weight of each evaluation aspect at the *L* + 1 layer is still *NW*_*i*_^*L*+1^ itself; that is,
    (18) $$\begin{array}{c} HW_{i}^{L+1}=NW_{i}^{L+1},\forall i=1,2,\ldots ,k. \end{array}$$
  (2) The integrated weight of each evaluation indication at the *L* + 2 layer is
    (19) $$\begin{array}{c} HW_{f}^{L+2}=NW_{i}^{L+1}\times NW_{f}^{L+2},\\ \forall i=1,2,\ldots ,k,\forall f=1,\ldots ,p;\cdots ;\forall f=1,\ldots ,q;\cdots ;\forall f=1,\ldots ,r. \end{array}$$

## 4. Empirical Study

### 4.1. Questionnaire Survey and Data Collection

The AHP expert questionnaire in this study employed 4 evaluation aspects and 16 evaluation indicators (see Table 2) in the pairwise comparison matrix. To ensure that the text and grammar of the AHP questionnaire were clear or check whether any important content concerning health promotion policies indicators was missing, this study invited three scholars and experts to conduct a pretest. After the text was revised twice by the experts and scholars, the formal AHP expert questionnaire was completed.

To evaluate the relative importance of the indicators, the formal AHP questionnaire survey was distributed among experts in different fields, including government personnel involved in Taiwan's health policy, experts and professors specializing in the field of health promotion, companies and private organizations that operate health promotion services for the elderly, and older adults among the general public.

AHP operating procedures were employed to assess the validity of the AHP questionnaire. If the consistency index (*CI*) value is less than or equal to 0.1, this means that a pairwise comparison matrix is consistent [15] and ensures that the experts' judgments are consistent and the questionnaire is valid. It should be noted that that the pairwise comparison matrix for each questionnaire should meet the requirements of consistency. If there is a pairwise comparison matrix that does not meet consistency requirements, this indicates that there is confusion in the experts' judgments. At this time, the experts must reassess this matrix until it meets the requirements of consistency.

A total of 48 questionnaires were distributed, and 44 valid questionnaires were recovered for an effective recovery rate of 92%. Robbins [57] suggested that the number of experts required for group decision-making problems should be 5–7 individuals. This indicates that the number of recovered valid questionnaires in this study was sufficient to provide representative opinions.

Table 4 contains basic information concerning the respondents who completed valid questionnaires. Men accounted for roughly 60% of respondents and women for roughly 40%. People between the ages of 51 and 60 accounted for one-half of the sample, and those over the age of 51 accounted for two-thirds of the sample. With regard to the level of education, approximately 40% of respondents had an undergraduate degree, while holders of master's and Ph.D. degrees each accounted for around 30%. In terms of professional background, roughly 25% each were, respectively, involved in business, academia, government, or were members of the general public.

### 4.2. Calculation Process and the Results

#### 4.2.1. Hierarchical Structure and the Code Names

To clearly express the subsequent calculation process, according to the hierarchical structure of Figure 1, each evaluation aspect and each evaluation indicator are represented by code names in parentheses, as follows:

1. Healthy living (*C*_1_): it includes “the promotion of personal health awareness and behavior (*C*_11_),” “well-planned health promotion plans for the elderly (*C*_12_),” “promotion of home medical services (*C*_13_),” and “seamless integration of medical services and social care (*C*_14_),” respectively.
2. Happy family (*C*_2_): it includes “training long-term care service personnel and providing professional medical care (*C*_21_),” “planning a family caregiver support service system (*C*_22_),” “promoting connection and mutual assistance between families and the community (*C*_23_),” and “guaranteeing the economic security of the elderly (*C*_24_),” respectively.
3. Vibrant society (*C*_3_): it includes “promotion of participation by older adults in work (*C*_31_),” “encouragement of the elderly to participate in voluntary service (*C*_32_),” “promotion of an education and learning system for older adults (*C*_33_),” and “encouragement of creative thinking concerning services for older adults (*C*_34_),” respectively.
4. Friendly environment (*C*_4_): it includes “the establishment of a network of continuous service resources (*C*_41_),” “establishment of community service resource centers (*C*_42_),” “creation of friendly living facilities and spaces (*C*_43_),” and “review of laws, regulations, and public education (*C*_44_),” respectively.

#### 4.2.2. Construction of a Fuzzy Positive Reciprocal Matrix

This study must construct 5 (1 + 4) pairwise comparison matrices. Due to the complicated calculation process of these pairwise comparison matrices and to save space, only the four evaluation aspects in the *L* + 1 layer are used to illustrate the calculation process of the fuzzy AHP method. As for the other 4 pairwise comparison matrices in the evaluation indicator layer, their calculation process is omitted because their calculation process is the same.

After ranking out 44 valid questionnaires, this paper compared the relative importance of the four evaluation aspects (*C*_1_–*C*_4_). This paper used the geometric mean method to integrate the opinions of experts and scholars (see Step 3 in Section 3.3) and calculate the triangular fuzzy numbers of the 4 evaluation aspects, as shown in Table 5.

Furthermore, according to the process of Step 4 in Section 3.3, this paper constructed a fuzzy positive reciprocal matrix, and the results are shown in Table 6.

#### 4.2.3. Calculating the Weights of Evaluation Aspects and Criteria for Each Layer

First, the data in Table 6 and the calculation process described in Step 5 to Step 8 in Section 3.3 were used to calculate the relative weights of the four evaluation aspects, as shown in Table 7.

Secondly, the normalized weight value (NW_*i*_^*L*+1^) calculated through the above steps is the value under the weight (A) column in Table 8. After that, the relative weights of each evaluation aspect and evaluation indicator can be calculated according to the above steps. Finally, this paper integrated the relative weights of each evaluation indicator to obtain the relative importance of each evaluation aspect and the evaluation indicator. The final summary result is shown in Table 8.

According to the data in Table 8, the important key indicators of health promotion policies for an aging society in Taiwan chiefly include the following:

(1) In terms of the evaluation aspects, the “healthy living” is the most important link in the health promotion policies of an aging society in Taiwan. Secondly, the “happy family” is considered the second most important link, the third is the “friendly environment,” and the fourth is the “vibrant society.”
(2) In terms of the evaluation indicators belonging to the four major evaluation aspects,
  1. In the aspect of the “healthy living,” the “promotion of personal health awareness and behavior” is the most important evaluation indicator.
  2. In the aspect of the “happy family,” the “guaranteeing the economic security of the elderly” is the most important evaluation indicator.
  3. In the aspect of the “vibrant society,” the “promotion of an education and learning system for older adults” is the most important evaluation indicator.
  4. In the aspect of the “friendly environment,” the “creation of friendly living facilities and spaces” is the most important evaluation indicator.
(3) Daniel [58] believes that industrial development must have two to six key factors that determine success. These key factors must be done very well for the industry to be successful. This paper used a total of 6 key evaluation indicators as the key factors in evaluating the health promotion policies for an aging society in Taiwan. The total weight of these six key indicators is 46.68%, accounting for about half of the overall weight. The results show that the most important six key indicators are the “promotion of personal health awareness and behavior (0.0883),” the “promotion of home medical services (0.0785),” the “guaranteeing the economic security of the elderly (0.0771),” the “planning a family caregiver support service system (0.0751),” the “well-planned health promotion plans for the elderly (0.0739),” and the “training long-term care service personnel and providing professional medical care (0.0739),” respectively.

### 4.3. Discussion

In this study, some discussions and suggestions are made concerning the foregoing six key indicators, as described in the following.

#### 4.3.1. Promotion of Personal Health Awareness and Behavior

This key indicator represents the most important factor influencing health promotion policies for Taiwan's aging society. Health promotion must start from individuals' health awareness, and the chief focus of health promotion is on guiding the elderly in taking care of their health. The goal of active health promotion for older adults is to instill a good attitude toward healthy living and good health awareness. Since good quality of life requires a healthy body, effective health-promoting behavior must become an everyday habit. Older adults must therefore rely on their individual daily health awareness to form habits of healthy behavior. To extend the healthy lifespans of older adults, methods including nutrition education, medication consultation, and regular exercise must be employed to enhance health awareness, which will cause older adults to be willing to participate in relevant health activities.

The experts and scholars in this study were consulted on how to promote personal health awareness and behavior and expressed that the government should set up learning systems for the elderly in local communities. The elderly can be provided with healthcare learning opportunities via education programs such as Evergreen College or schools for older adults. In addition, health concepts can be publicized using marketing approaches and multimedia systems spanning TV, radio, the Internet, video, and other methods. The establishment of community fitness clubs will allow the elderly to develop the beneficial habit of exercising every day. Educational institutions throughout the country should provide internships for medical college students interested in education for the elderly. This education, which may be administered through the community or home education, can encompass the aspects of a balanced diet, a healthy lifestyle, and quitting smoking and alcohol.

Health-related government agencies can arrange regular health check-ups, medical and health consultations, and psychological consultations for older adults. During the post-COVID-19 pandemic, it is necessary to actively strengthen correct disease prevention concepts. The elderly should be educated in the prevention of the pandemic, the importance of vaccinations, the importance of wearing masks, regularly checking their temperature, washing hands before and after meals, disinfection with alcohol-based solutions, reducing touching eyes, mouth, and nose, and avoidance of crowded places. These practices will help older adults to establish correct personal protection concepts, which will help fulfill the goals of healthcare and health promotion.

#### 4.3.2. Promotion of Home Medical Services

This key indicator is the second most important factor influencing health promotion policies for Taiwan's aging society. The basic preconditions for acceptance as home medical care recipients are either difficulty of leaving home, disability, or disease and must have been assessed by doctors as having definite medical needs. Home medical care integrates care systems in the five areas of medical care, nursing care, life support, health prevention, and home living. It should also have the goal of allowing older adults with physical disabilities to continue to live in their original areas. Appropriate medical care should be provided by the local area through the establishment of community-based medical services, and community resources in cross-professional fields should be integrated. These measures will create an environment and linkage that will benefit family and community health and provide patients with comprehensive medical and life care. The promotion of home medical services will therefore be very important.

The experts suggested that home care teams can be formed to provide medical services to older adults, which will reduce the burden on family members taking care of elderly relatives. In particular, home medical care services will be of great importance to health promotion among the unhealthy elderly. The government should strengthen attention to rural areas and areas with insufficient medical resources, actively integrate regional health and medical capabilities, allocate adequate medical budgets, and form medical project teams (including doctors, pharmacists, nursing staff, social workers, and psychologists). The government should further plan and arrange doctor consultations, drug prescriptions, health checks, medical consultations, nursing care, and psychological consultations as elements of home medical services. These services can assist older adults in a postacute stage or with disabilities to return to their homes with peace of mind and further strengthen continuous medical care. Apart from enabling the elderly to recover in less time, this will also ensure that older adults can receive effective medical protection and maintain a good quality of life. In addition, it will allow the elderly with mobility difficulties to receive comprehensive home medical services and achieve the ideals of health promotion for an aging society.

#### 4.3.3. Guaranteeing the Economic Security of the Elderly

This key indicator is the third most important factor affecting health promotion policies for Taiwan's aging society. Due to changes in the social environment and the continued decline in household senior care functions, as well as continued demographic aging and the acceleration of the decline in birthrates, many older adults hope their future economic life should not cause trouble and stress for their children. Many older people in Taiwan have unstable financial resources, resulting in a poor quality of life in their later years. The government provides elderly allowances to the less-privileged, but the effect of these is still quite limited. Taking care of the physical and psychological needs of the elderly and enabling them to spend their twilight years in peace and comfort is a major challenge for the government. Strengthening the social security of the elderly security system, establishing a feasible and complete economic security guarantee system, and helping people in making proper financial and economic preparations for their older years are some of the challenges faced by Taiwan's society.

The experts and scholars noted that people should be prepared mentally for their old age at an early date and preferably at the beginning of their old age. Building the soft power of personal economy and planning financial savings should be encouraged as preparations for old age. Secondly, government policies should strengthen economic security for the elderly, such as through education concerning social insurance and financial planning for retirement. Lastly, government policies should strengthen the planning of protection, healthcare, residential safety, material supply, and a safe environment for the elderly. The government should develop a sound and sustainable social insurance system and improve the economic security of the elderly through policy, implementation of a national pension system, protection of existing pension systems for the elderly, and implementation of long-term insurance. This will reduce the economic risks faced by the elderly and ensure that the elderly can enjoy economic stability, peace of mind, and healthy and happy retirement life.

#### 4.3.4. Planning a Family Caregiver Support Service System

This key indicator is the fourth most important factor influencing health promotion policies for Taiwan's aging society. In earlier days, society in Taiwan was under the influence of the traditional family system, in which the elderly were supported by their families, and their care was a family responsibility. This system remained a cornerstone of social stability for a long time. But with urbanization, family members spend less time at home due to work needs, and gender equality and the increase in women's employment have also caused changes in the traditional family division of labor. This has led to insufficient family caregiving manpower and increased care burdens. The long-term care system has been growing more diversified and now includes institutional daycare, community-based care, home-based care, and care by family members. To meet care needs, allow family caregivers “off time,” and reduce the pressure and burden on family caregivers, the government should actively establish a family caregiver support system. To establish comprehensive family caregiver service resources, the government should deploy care resources through policies and provide relevant support services. This will improve the quality of care services for the elderly and ensure that both caregivers and recipients of care are helped.

The experts and scholars indicated that planning a family caregiver support service system has become an important issue. Family caregivers commonly complain of excessive care workloads and the need to bear heavy physical, psychological, emotional, and time burdens. The caregivers facing such heavy burdens hope to receive assistance from outside the home. The government should therefore integrate existing family caregiver support services and strengthen the administrative capacities of family caregiver support services. The goal of this effort should be to gradually establish a social and psychological support network for family caregivers. With the rapid increase in the demand for senior care, the family caregiver support service system is becoming more important, and government agencies should develop various alternative care services as quickly as possible. These alternative services may consist of daytime care centers, elderly care centers, family care centers, and community care bases. Such alternative care services will provide family caregivers with opportunities for rest and allow the older adults being cared for to receive the highest quality professional healthcare.

#### 4.3.5. Well-Planned Health Promotion Plans for the Elderly

This key indicator is the fifth most important factor influencing health promotion policies for Taiwan's aging society. In line with the rapid aging of the population, the government should investigate the physical, mental, and social life of the elderly and should strive to monitor and control the risk factors for various chronic diseases. The government should develop health promotion intervention plans suitable for older adults via research. Various health promotion activities can then be employed to carry out preventive health education advocacy and various measures geared to helping older adults to adopt healthy lifestyles.

The experts and scholars noted that government should actively initiate general surveys of the health status of the elderly, which will allow assessment of older adults' health status distribution or classification. Suitable health promotion programs based on the physical and mental health status of the elderly can then be introduced. Such programs may focus on fitness exercises, physical training, outdoor activities, and study visits for the healthy elderly and will improve the fitness and vitality of participants. “Rehabilitation” training plans can be developed for older adults with suboptimal health and should seek to help them regain their normal health condition. For nonhealthy older adults, a comprehensive medical care policy can be formulated and deployed through home medical services. In the case of older adults living alone, the government should actively address their health and living conditions, including dietary nutrition, material supply, exercise awareness, vaccination, and regular health check-ups. Care centers can be established in the community, and borough and neighborhood chiefs should pay close attention to the living conditions of the elderly in order to prevent accidents, falls, and lonely deaths.

#### 4.3.6. Training Long-Term Care Service Personnel and Providing Professional Medical Care

This key indicator is the sixth most important factor influencing health promotion policies for Taiwan's aging society. Aging is inevitable. Coupled with the rapid changes in modern society, many family members are not as close to each other as in the traditional society of the past and may be isolated or estranged. The government must use more channels to let the members of the younger generation understand that aging is natural and that younger individuals should be more empathetic and understanding and have a friendly attitude toward older adults. Young people should also have positive perceptions of care services for the elderly. This will ensure that new generations understand the process of aging and the needs of older adults from an early age. It is hoped that interaction between different generations will enhance mutual understanding among the young and establish close intergenerational connections. This will also help younger individuals to realize the value of the elderly, and continuity of family affection, and the importance of reciprocity. It is not easy to realize these ideals at present, however. This is because Taiwan is short of manpower for long-term care services, and there is a lack of effective education and policy integration. As a result, all sectors of society fail to correctly perceive the nature of the work of caring for the elderly. Existing incorrect perceptions have reduced the willingness of people to get involved in long-term care for older adults. Moreover, the hard work, poor benefits, low salaries of long-term care service personnel, and the need to improve their professional image have hindered the commitment of manpower and talent to this industry. As a result, there is currently insufficient care service staff. Since long-term care services require not only manpower but also the talent needed to promote the progress and development of this industry, government policies should be geared to improving the salaries and benefits of care service providers. This will ensure care service providers' economic stability and related labor benefits and thereby increase the flow of manpower and talent into long-term care.

The experts suggested that, with the coming of a superaged society in Taiwan, many elderly people with poor health will need service personnel to provide professional medical care. To train professional service personnel, the government should actively introduce various types of training and strive to overcome manpower shortages through manpower training strategies geared to its long-term care development policy. In addition, long-term care service personnel should be cultivated through the diversification of functional agencies. Good medical care for the elderly can only be provided via the development of professional medical curricula. The government should focus on the serious problem of insufficient human resources and actively cooperate with the school education system to designate long-term care as a formal internship course for departments such as nursing. Universities and junior colleges should pay greater attention to long-term care and medical nursing, and qualifications in these fields can be included in national certification examinations. Colleges and universities can be directed to improve the training of long-term care professionals, and it will be necessary to plan professional certification for long-term care personnel. Active planning of professional medical training for caregivers and encouraging the improvement of their professional competence will also be very important. This study looks forward to the government's meeting current long-term care needs through the training of long-term caregivers, measures to reduce the psychological burden on family caregivers, the promotion of family well-being, and other efforts to achieve the goal of health promotion in an aging society.

## 5. Concluding Remarks

Taiwan's aging population is increasing rapidly. In the face of changes in social values and lifestyles, the burden of family care is gradually increasing, and the formulation of health promotion policies has grown steadily more important. Discussion of factors affecting the development of health promotion in an aging society will shed light on the needs of the elderly and also point out the health promotion strategies that should be prioritized in view of the government's limited resources. Evaluation of the key indicators of Taiwan's health promotion policies is therefore an important research topic.

To provide policy implementation stakeholders with a reference for health promotion policies aimed at the elderly, this study used the fuzzy AHP method to empirically analyze key indicators of health promotion policies for Taiwan's aging society. This study also assessed the priority of key indicators of health promotion policies. Important factors affecting the development of health promotion policies were obtained from a review of the literature and expert opinions. These factors included four major evaluation aspects and 16 evaluation criteria. An AHP expert questionnaire was then issued to major policy evaluation stakeholders. After the fuzzy AHP method was used to find the relative weights of each evaluation aspect and each indicator, this study made the following empirical findings: (1) “Healthy living” was the most important evaluation aspect of health promotion policies for Taiwan's aging society. (2) The top six key indicators of health promotion policies for Taiwan's aging society were “promotion of personal health awareness and behavior,” “promotion of home medical services,” “guaranteeing the economic security of the elderly,” “planning a family caregiver support service system,” “well-planned health promotion plans for the elderly,” and “training long-term care service personnel and providing professional medical care,” respectively.

Lastly, this paper discusses the management implications of its research findings concerning health promotion policies for government agencies, academic institutions, industry, and older members of the public.

With regard to government agencies, since demographic aging is a major issue of concern to all countries' governments, industry, government, academia, and the public must work in close coordination to develop feasible care policies for Taiwan's aging population. The six key indicators found in this study can enable government agencies to quickly and clearly formulate relevant health promotion strategies. We look forward to the joint efforts of the government, the public, and all parts of society to summon the capabilities of the private sector for the purpose of health promotion. This campaign will call on local charitable organizations, private companies, public interest groups, and charitable foundations to commit their financial resources and resources to assist with the implementation of relevant policies and measures. Because of this, we hope that the government will take our recommendations concerning this study's key indicators as an administrative reference and strive to help older adults enjoy physical and mental health and harmonious lives in old age through the promotion of health functions and capabilities.

With regard to academia, the findings of this study indicate that the development of academic programs should consider incorporating whole-person health promotion education and provide training in health functions and behavior. This will facilitate the maintenance of highly effective health promotion behavior from childhood to old age. In addition, we believe that the six key indicators will facilitate the setting of clearly defined health promotion development goals for the training of long-term care personnel and medical professionals.

With regard to industry, medical and technological progress have enabled the steady lengthening of people's life expectancy. This trend toward longer lives has also given rise to various aging industries, and we can foresee that health promotion and healthcare industries for older adults will continue to flourish in the future. As a consequence, how to achieve even better service quality and ensure the industry's sustainable development will be an important future issue. We expect that the six key indicators will enable the health promotion and healthcare industry to better understand the various future needs of the health promotion market and help managers to achieve greater effectiveness.

In the case of older adults, a superior care service system will ensure that the needs of every person entering old age will be the most urgent needs. According to statistics from the Taiwan Bureau of National Health Insurance, there has been steady annual growth in health insurance reimbursements, which indicates that, due to factors such as living habits, attitudes, living environment, diet, and stress, a growing number of people suffer from chronic disease and require medical intervention. We therefore believe that this study's six key indicators have real reference value toward health promotion and care, can help ensure that older adults and family members make the best use of medical resources, and can guide the establishment of healthcare approaches that can save time, effort, and resources.

Furthermore, as for this study's academic contribution, because Taiwan is currently fighting the COVID-19 pandemic, disease prevention is the most important health focal point. Nevertheless, as the pandemic gradually recedes, the focus of health administration will inevitably shift to health promotion policies and measures. Based on our empirical analysis, to effectively implement health promotion for Taiwan's aging society, we recommend that the six key indicators found in this study be taken as the leading focal points of health promotion policies meeting the needs of Taiwan's future superaged society. In addition, this study relied on rigorous empirical analysis and expert questionnaire interviews to assess key indicators of health promotion policies. During this time of health promotion and healthcare development, the findings of this study can provide both theoretical value and practical recommendations concerning the government's policies, academic institutions' planning of education and training, and the industry's development.

## Figures and Tables

**Figure 1:** Hierarchical structure diagram.

**Table 1:** Preliminary health promotion policy development indicators.

Authors indicators	A	B	C	D	E	F	G	H	I	J	K	L	M	N	O	P	Q	R
Promotion of personal health awareness and behavior	✓	✓	✓	✓		✓	✓		✓	✓							✓	✓
Well-planned health promotion plans for the elderly		✓	✓	✓			✓		✓	✓	✓					✓	✓	✓
Promotion of home medical services				✓		✓	✓		✓							✓		✓
Seamless integration of medical services and social care			✓	✓		✓	✓									✓		✓
Training long-term care service personnel and providing professional medical care				✓			✓				✓	✓				✓	✓	✓
Planning a family caregiver support service system				✓	✓	✓	✓	✓								✓		✓
Promoting connection and mutual assistance between families and the community			✓	✓		✓	✓	✓					✓					✓
Guaranteeing the economic security of the elderly				✓		✓	✓		✓	✓	✓	✓				✓		✓
Promotion of participation by older adults				✓	✓	✓					✓	✓				✓		
Encouragement of the elderly to participate in voluntary service			✓	✓		✓	✓				✓							✓
Promotion of an education and learning system for older adults				✓		✓	✓										✓	✓
Encouragement of creative thinking concerning services for older adults			✓	✓		✓					✓							✓
Establishment of a network of continuous service resources				✓		✓					✓	✓	✓			✓		✓
Establishment of community service resource centers		✓		✓							✓	✓				✓		✓
Creation of friendly living facilities and spaces			✓	✓		✓								✓	✓			✓
Review of laws, regulations, and public education		✓		✓		✓										✓	✓	✓

Note: A: Kao et al. [3]. B: WHO [12]. C: Hsu and Hu [16]. D: HPA [18]. E: Tadić et al. [20]. F: Liao [21]. G: Bonder and Bello-Haas [24]. H: Liimatainen et al. [27]. I: ODPHP [31]. J: Gatz et al. [32]. K: Chen [33]. L: Haber [34]. M: Colello and Napili [35]. N: Anderson et al. [36]. O: Putnam [37]. P: Lee et al. [38]. Q: Suzuki [39]. R: Feng [40]

**Table 2:** Preliminary indicators of health promotion policies for Taiwan's aging society.

Aspects	Indicators	Explanation
Healthy living	Promotion of personal health awareness and behavior	Improvement of older adults' oral, physical, psychological, and social health concepts. Promotion of self-care behavior for the purpose of prolonging the lifespan of the elderly. Strengthening awareness of healthy diet and nutrition, smoking cessation, medication, exercise, and regular living habits. Improvement of the health awareness of older adults and promotion of healthy behaviors.
	Well-planned health promotion plans for the elderly	Planning of health promotion policies and plans aimed at older adults, including plans focusing on diet and nutrition, oral healthcare, exercise skills, and mental health. Refinement of various medical service strategies for older adults. Use of health promotion activity programs to improve the self-care and health capabilities of the elderly.
	Promotion of home medical services	Promotion of home medical services using home care teams. Provision of integrated community medical services. Assisting older adults needing postacute care or with disabilities to return to their homes. Provision of friendly medical services for the elderly, strengthening continuous care, and ensuring healthy living for the elderly.
	Seamless integration of medical services and social care	Connecting the postacute care, community rehabilitation, and long-term care systems using information technology. Constructing a comprehensive, convenient continuous care system so that older adults and their family members can live healthy lives at home with peace of mind after breaks in medical care.

Happy family	Training long-term care service personnel and providing professional medical care	Actively introducing various types of training concerning long-term care services. Providing dual-track training of long-term care personnel through vocational training and school education. Planning and developing a professional grading system for long-term care personnel. Developing a diversified manpower portfolio and providing professional healthcare to older adults in order to relieve family members' psychological pressure. Offering sustainable long-term care services and promoting family well-being.
	Planning a family caregiver support service system	With the goal of improving the overall well-being of older adults and their families, planning an active family caregiver support service system to enhance the connection and integration between older adults and their family members, which will effectively ease families' care burden and enhance their overall well-being.
	Promoting connection and mutual assistance between families and the community	Planning of family-centered policies in response to changes in household structure and social values, design of innovative activities promoting interaction between the elderly and other family members, promotion of communication between generations, strengthening of cooperation between families and the community, and facilitation of community mutual care for older adults.
	Guaranteeing the economic security of the elderly	Improving economic security protection mechanisms and the pension system for the elderly. Establishment of knowledge concerning financial management and insurance planning for the elderly, which will allow the sharing and reduction of the economic risks and enable older adults to enjoy economic stability and a worry-free and healthy retired life.

Vibrant society	Promotion of participation by older adults	Active promotion of participation by the elderly in work and provision of a friendly environment for elderly employment. Appropriately adjusting working hours, work content, and working format in accordance with the age and health status of older employees and alleviation of the physical and mental health effects of the rapid change in older adults' roles after retirement.
	Encouragement of the elderly to participate in voluntary service	Avoiding the impact of retirement on older adults' daily activities. Promotion of retirement preparation education and services for the elderly. Helping the elderly to actively plan their retirement lives and encouraging their participation in volunteer service intended to give back to society. Developing diverse innovative service model for volunteers, with the goal of slowing the aging process and promoting health.
	Promotion of an education and learning system for older adults	Application of the flipped classroom concept. Integration of the lifelong learning education system. Comprehensive promotion of training for older adult education professionals. Establishment of professional qualification certification for senior citizens. Encouragement of older adults to contribute their wisdom and pass on their experience by becoming teachers and encouragement of lifelong learning so that the elderly can continue to learn while growing old and achieve the goal of active aging.
	Encouragement of creative thinking concerning services for older adults	Encouragement of innovative service thinking geared toward the demands of older adults. Active investment in the development of the equipment, products, and services required to meet the food, clothing, housing, transportation, and entertainment needs of an aging society and satisfying the current and future living and health promotion needs of older adults.

Friendly environment	Establishment of a network of continuous service resources	Connection of different types of information, materials, goods, and services through the Internet of things and the Internet. Connection of local physical payment services to form a comprehensive resource network providing services. Satisfying the diversified service needs of the future's aging society and promoting healthcare.
	Establishment of community service resource centers	Building hubs integrating resource networks to provide convenient and safe living for the elderly. Establishing integrated community service resource centers. Establishing comprehensive community resources allowing older adults to age in place. Ensuring personal safety and improving medical care for the elderly.
	Creation of friendly living facilities and spaces	Promoting mechanisms ensuring that public construction better serves older adults. Comprehensive review and revision of relevant laws and regulations governing buildings, spatial design, and housing. Promoting senior-friendly public transportation facility spaces and environments (including software and hardware amenities and equipment) and creating senior-friendly living environments.
	Review of laws, regulations, and public education	Comprehensive review and amendment of relevant laws and regulations in order to eliminate age discrimination and barriers so that society as a whole has a more positive understanding and acceptance of older adults and helps older adults enjoy healthy aging. Use of the national compulsory education and public education system to instill a positive understanding of and respect for the elderly among the public.

Source: author's comprehensive collation.

**Table 3:** Saaty scale, definition, and explanation.

Saaty scale	Definition	Explanation
1	Equal importance	The contribution of the two plans is of equal importance equally
3	Slightly importance	Experience and judgment tend to favor a certain plan slightly moderately
5	Essential importance	Experience and judgment tend to favor a certain plan strongly
7	Demonstrates importance	A very strong preference is shown for a certain plan demonstratively
9	Absolute importance	There is enough evidence to favor a certain plan extremely
2, 4, 6, 8	Intermediate values of adjacent scales	When a compromise value is needed

**Table 4:** Profiles of the group experts.

Basic information	Distribution	Number of experts	Percentage (%)
Gender	Male	26	59.09
	Female	18	40.91
	Total	44	100

Age	36–40	4	9.09
	41–45	4	9.09
	46–50	7	15.91
	51–55	12	27.27
	56–60	10	22.73
	Over 61	7	15.91
	Total	44	100

Education	Bachelor	18	40.91
	Master	14	31.82
	PhD	12	27.27
	Total	44	100

Professional background	Governments	11	25
	Scholars	11	25
	Companies	11	25
	General elderly	11	25
	Total	44	100

**Table 5:** Triangular fuzzy numbers of the 4 evaluation aspects.

Evaluation aspect	Triangular fuzzy number	Evaluation aspect
*C*_1_	(0.143, 1.287, 7.0)	*C*_2_
*C*_1_	(0.20, 3.311, 8.0)	*C*_3_
*C*_1_	(0.143, 2.972, 8.0)	*C*_4_
*C*_2_	(0.250, 3.134, 7.0)	*C*_3_
*C*_2_	(0.250, 2.444, 8.0)	*C*_4_
*C*_3_	(0.20, 0.664, 7.0)	*C*_4_

**Table 6:** Fuzzy positive reciprocal matrix of the four evaluation aspects.

	*C*_1_	*C*_2_	*C*_3_	*C*_4_
*C*_1_	(1, 1, 1)	(0.143, 1.287, 7.0)	(0.20, 3.311, 8.0)	(0.143, 2.972, 8.0)
*C*_2_	(0.143, 0.777, 7.0)	(1, 1, 1)	(0.250, 3.134, 7.0)	(0.250, 2.444, 8.0)
*C*_3_	(0.125, 0.302, 5.0)	(0.143, 0.319, 4.0)	(1, 1, 1)	(0.20, 0.664, 7.0)
*C*_4_	(0.125, 0.336, 7.0)	(0.125, 0.409, 4.0)	(0.143, 1.506, 5.0)	(1, 1, 1)

**Table 7:** Calculation process of relative weights of the four evaluation aspects.

	*C*_1_	*C*_2_	*C*_3_	*C*_4_
${\tilde{Z}}_{i}^{L+1}$	(0.253, 1.886, 4.601)	(0.307, 1.562, 4.450)	(0.244, 0.503, 3.440)	(0.217, 0.675, 3.440)
${\tilde{W}}_{i}^{L+1}$	(0.016, 0.408, 4.502)	(0.019, 0.338, 4.354)	(0.015, 0.109, 3.366)	(0.014, 0.146, 3.366)
$G\left({\tilde{W}}_{i}^{L+1}\right)$	1.025	0.954	0.636	0.660
NW_*i*_^*L*+1^	0.313	0.291	0.194	0.202

**Table 8:** The integration weights of evaluation aspects and evaluation indicators.

Evaluation aspect	Weight (A)	Evaluation indicator	Weight (B)	Integration weight (C) = (A)∗(B)
Healthy living (*C*_1_)	0.313 (1)	Promotion of personal health awareness and behavior (*C*_11_)	0.282 (1)	0.0883 (1)
		Well-planned health promotion plans for the elderly (*C*_12_)	0.236 (3)	0.0739 (5)
		Promotion of home medical services (*C*_13_)	0.251 (2)	0.0785 (2)
		Seamless integration of medical services and social care (*C*_14_)	0.231 (4)	0.0723 (7)

Happy family (*C*_2_)	0.291 (2)	Training long-term care service personnel and providing professional medical care (*C*_21_)	0.254 (3)	0.0739 (5)
		Planning a family caregiver support service system (*C*_22_)	0.258 (2)	0.0751 (4)
		Promoting connection and mutual assistance between families and the community (*C*_23_)	0.223 (4)	0.0649 (8)
		Guaranteeing the economic security of the elderly (*C*_24_)	0.265 (1)	0.0771 (3)

Vibrant society (*C*_3_)	0.194 (4)	Promotion of participation by older adults in work (*C*_31_)	0.231 (3)	0.0448 (14)
		Encouragement of the elderly to participate in voluntary service (*C*_32_)	0.270 (2)	0.0524 (12)
		Promotion of an education and learning system for older adults (*C*_33_)	0.273 (1)	0.0530 (11)
		Encouragement of creative thinking concerning services for older adults (*C*_34_)	0.226 (4)	0.0438 (15)

Friendly environment (*C*_4_)	0.202 (3)	Establishment of a network of continuous service resources (*C*_41_)	0.245 (3)	0.0495 (13)
		Establishment of community service resource centers (*C*_42_)	0.276 (2)	0.0557 (10)
		Creation of friendly living facilities and spaces (*C*_43_)	0.281 (1)	0.0568 (9)
		Review of laws, regulations, and public education (*C*_44_)	0.198 (4)	0.040 (16)

*Note.* The parentheses after the weight number mean the ranking.

## Data Availability

The data used to support the findings of this study are included within the article.
